# A Lightweight CNN Model Based on GhostNet

**DOI:** 10.1155/2022/8396550

**Published:** 2022-07-31

**Authors:** Zhong Wang, Tong Li

**Affiliations:** School of Computer Science and Technology, Hefei Normal University, Hefei 230601, China

## Abstract

The existing deep learning models have problems such as large weight parameters and slow inference speed of equipment. In practical applications such as fire detection, they often cannot be deployed on equipment with limited resources due to the huge amount of parameters and low efficiency. In response to this problem, this paper proposes a lightweight smoke detection model based on the convolutional attention mechanism module. The model is based on the YOLOv5 lightweight framework. The backbone network draws on the GhostNet design idea, replaces the CSP structure of the FPN and head layers with the GhostBottleNeck module, adds a convolutional attention mechanism module to the backbone network layer, and uses the CIoU loss function to improve the regression accuracy. Using YOLOv5s as the benchmark model, the parameter amount of the proposed lightweight neural network model is 2.75 M, and the floating-point calculation amount is 2.56 G, which is much lower than the parameter amount and calculation amount of the benchmark model. Tested on the public fire dataset, compared with the traditional deep learning algorithm, the model proposed in the paper has better detection performance and the detection speed is significantly better than the benchmark model. Tested under the unquantized simulator, the speed of the proposed model to detect a single picture is 60 ms, which can meet the requirements of real-time engineering applications.

## 1. Introduction

In 2021, a total of 748000 fires were reported in China, including 1987 deaths, 2225 injuries, and 6.75 billion yuan in direct property losses. In 2020, a forest fire in Yunnan burned for three days and nights. The area of the fire reached 170 hectares, and 5800 people were involved in suppressing the fire. In addition, a bush fire in Australia burned for more than four months, burning an area of 170000 square kilometers and resulting in the loss of many vegetation and animals. The smoke generated by the fire poured into the stratosphere, and the impact cannot be fully restored for a long time [1]. Fire not only seriously threatens the safety of human life but also has a great effect on the ecological environment. Fire prevention is very important to protect people's lives and property and has important scientific research significance [2, 3].

Traditional fire detection technologies include contact-type fire detectors such as temperature detectors [4] and smoke detectors [5, 6], which are commonly used in most public places. However, the disadvantages of this kind of detector are limited to indoor detection, aging, alarm time delay, etc. Thus, it is difficult to carry out fire monitoring in outdoor spaces. Compared with traditional contact fire detectors, noncontact video fire detection technology has the characteristics of fast response, wide detection range, and low hardware cost and is suitable for fire monitoring in large indoor and outdoor spaces and forests. Video fire detection technology can be divided into flame detection [7] and smoke detection [8] according to the detection object. Generally, in the early stages of a fire, the smoke appears earlier than the flame and is not easy to cover, and the flame will only be generated in the middle of the fire. When the flame is detected, the fire has occurred, which makes it impossible to prevent and control it for the first moments. Therefore, the current video fire detection technology mainly focuses on detecting smoke.

Smoke detection technologies include traditional machine learning-based methods and deep learning-based methods. The smoke detection technology based on traditional machine learning includes two parts: feature extraction and classifier design. The core research is smoke feature research. Commonly used smoke features mainly include artificially designed features such as the color [9], texture [10], motion [11], background contrast [12], and combinations of various features [13]. Smoke detection technology based on traditional machine learning has difficulty meeting the application requirements of real-time detection in terms of accuracy and false alarm rate. With the successful application of deep learning technology in the field of computer vision, deep convolutional neural networks are widely used in smoke detection. At present, smoke detection algorithms based on deep learning are mainly divided into two categories. One is a two-stage target detection model based on region extraction, such as R-CNN (regions convolutional neural network) [14–16], Fast R–CNN [17], and Faster R–CNN [18], which divide the target detection into the following two steps: feature extraction and feature classification. The other category is a one-stage target detection model that directly performs location regression, such as the SSD (single-shot multibox detector) [19] and YOLO (you only look once) [20] series, which converts target detection into a regression problem.

Most smoke detection algorithms based on deep learning rely on convolutional networks for feature extraction. To solve the problems of efficiency and storage, researchers adopt network pruning [21], network parameter quantization [22], and knowledge distillation [23] and design lightweight networks to improve the speed of inference. For example, MobileNet v1-v3 [24–26] and EfficientDet [27] were proposed by Google, GhostNet [28] was proposed by Huawei, and ShuffleNet [29, 30] and SqueezeNet [31] were proposed by Megvii. These networks are well constructed. It can reduce the number of model parameters and improve the accuracy of the network detection, which plays an important role in real-time smoke detection.

Although smoke detection technology has been widely used, the smoke detection scene is complex and changeable, and the accuracy and robustness of the existing technology in complex smoke scenes still have difficulty meeting the needs of popularization and application. Therefore, this paper designs a lightweight network based on the YOLOv5 framework, draws on the design ideas of GhostNet, and adds the CBAM attention mechanism [32] to achieve model compression and speed up inference without reducing the accuracy of the model. This model greatly reduces the need for hardware environment and uses MNN as the framework for unquantified testing. The specific work is as follows:

1. Improve the focus structure to reduce the parameters and calculation amount of the focus layer.
2. The backbone network adopts the GhostNet module, and the CSP of the FPN and the head layers is modified to a Ghost bottleneck.
3. Add an attention mechanism CBAM to the backbone network layer.

The rest of the paper is arranged as follows: Section 2 introduces the work related to smoke detection; Section 3 focuses on the description of lightweight smoke detection models and implementation details; Section 4 compares the performance of different smoke detection models on smoke detection datasets; finally, a summary and outlook are given.

## 2. Related Works

Traditional smoke detection technology tries to obtain the characteristics of smoke to distinguish from other interfering substances and performs smoke detection by manually setting the smoke characteristics, but the detection rate and false alarm rate have difficulty meeting the application requirements. With the application of deep learning techniques in the field of computer vision [33–35], researchers have used deep convolutional neural networks for smoke detection [36–39], which can learn deeper feature models. Luo et al. [40] combined convolutional neural networks with traditional foreground extraction methods for smoke detection, extracted suspected smoke regions based on motion and color information, and used a CNN to extract regional features for classification. Pundir and Raman [41] input texture features into deep belief texture learning to train the smoke recognition model. Zhang et al. [42] solved the problem of insufficient sample data by inserting real smoke images in the forest background and adopted Faster R-CNN to detect wildland forest fire smoke. Filoneko et al. [43, 44] adopted classical convolutional neural networks (including AlexNet, Inception-V3, Inception-V4, ResNet, VGG, and Xception) to conduct experimental verification on four large-scale smoke image databases. Sharma et al. [45] used two pretrained deep convolutional neural networks, VGG and ResNet50, to test unbalanced datasets and found that deeper CNNs performed better on more challenging datasets. Yin et al. [46] proposed a 14-layer deep normalization and convolutional neural network (DNCNN) to achieve automatic feature extraction and classification. To further reduce the problem of model overfitting caused by insufficient training samples, more training samples are generated from the original training set by using various data enhancement techniques. Muhammad et al. [47] proposed an energy-saving edge-assisted smoke detection method based on a deep convolutional neural network for foggy monitoring scenes, and the early smoke detection methods outperformed the state-of-the-art methods. Xu et al. [48] proposed a new video smoke detection method based on a deep saliency network, which uses a circular convolutional structure to construct a pixel-level saliency detection network and uses the fused features for saliency reasoning. Li et al. [49] proposed extracting suspicious smoke regions by smoke region proposal, pruning and reconstructing a convolutional neural network to improve real-time detection, and proposing a regularized loss function called score clustering to improve the accuracy of the model. Liu et al. [50] proposed a two-stage smoke detection method. In the first stage, block DNCNN is used to detect the suspicious smoke area from each frame image and put forward the concept of visual change image. In the second stage, the SVM classifier is used to classify the HOG features of the visual change image of the suspected smoke area.

Although smoke detection technology based on deep learning has achieved good results, with the improvement of the performance of the smoke detection algorithm, the number of convolutional layers also increases, resulting in the problems of large weight parameters and slow equipment reasoning speed. In practical applications, it is often unable to be deployed on equipment with limited resources because of the high parameter quantity and low efficiency. To solve the problem of efficiency and storage, researchers have designed lightweight networks to improve the inference speed. For example, the YOLOv3-Tiny [51] network launched for high parameters and inference speed is a simplified version of the YOLOv3 network. Iandola et al. [52] proposed SqueezeNet. The main idea is to replace the 3 × 3 convolution with a 1 × 1 convolution and reduce the amount of computation and parameters by reducing the number of channels of the 3 × 3 convolution. Howard et al. [53] proposed MobileNet, which mainly uses many neural networks designed with depthwise separable convolutions, which can greatly reduce the number of parameters and computations. MobileNetv2 employs a reverse residual block, while MobileNetv3 achieves better performance with fewer floating-point numbers. Based on MobileNetv3, GhostNet [54] adopts an inexpensive linear operation method to obtain richer output feature maps at a lower cost of model parameters to increase the feature extraction capability to solve the redundancy of feature maps. Zhang et al. [55] proposed ShuffleNet, which uses group convolution and channel shuffling operations to effectively reduce the computational complexity of point convolution and achieve superior performance. ShuffleNetV2 further considers practical speed in compact model design. In the field of smoke detection, Silva et al. [56] proposed a novel lightweight CNN model through RGB images, which can be used from aerial images of UAVs and video surveillance systems and combined with edge computing equipment to process images through a convolutional neural network. Pan et al. [57] used weakly supervised fine segmentation and lightweight Faster R–CNN to propose a collaborative area detection and classification framework for fire smoke, which can simultaneously achieve early warning, area detection, and classification of fire smoke. To reduce the complexity of Faster R–CNN, this method introduces knowledge distillation technology to compare the structure of the model. With the advancement of mobile devices and the diversified development of application scenarios, lightweight networks show higher engineering value. This paper balances between the accuracy and speed of the model, reasonably optimizes the YOLOv5 model, and designs a lightweight improved model based on the GhostNet and CBAM attention mechanisms. Without reducing the accuracy of the model, it realizes model compression and improves the reasoning speed, which greatly reduces the dependence on the hardware environment.

## 3. Methodology

### 3.1. YOLOv5

YOLO (you only look once) is widely used as a general object detection model. YOLOv1 uses one stage to complete the classification and positioning of objects, and then YOLOv2 [58] and YOLOv3 [59] further improve the speed and accuracy to accelerate object detection in the industrial world. YOLOv4 [60] can achieve training on an ordinary GPU. Currently, the YOLO series has developed into YOLOv5. Compared with YOLOv4, YOLOv5 is more flexible. To some extent, the YOLOv5 model is the most state of the art of all the known YOLO series. It provides four versions in the following ascending sizes: YOLOv5s, YOLOv5m, YOLOv5l, and YOLOv5x. The model size and accuracy of the four versions increase in turn and are distinguished by the number of bottlenecks. The channel and layer control factors are used to realize the version change, and the appropriately sized model can be selected according to the application scenario. This paper mainly implements model compression and acceleration, making it easier to apply to the embedded devices with limited resources. Therefore, YOLOv5s is used as the benchmark model with the smallest network depth and feature map width. YOLOv5s is mainly composed of the backbone and head. The backbone includes the focus, C3, and SPP modules, and the head includes the neck and detect modules for extracting fusion features.

### 3.2. Lightweight YOLOv5

Compared with the traditional YOLOv5s, this paper first gives the implementation method of some modules. The main improvements include the Focus_mod module, the GBN module (Ghost bottleneck), and the attention mechanism CBAM. The specific details are presented in the following subsections.

#### 3.2.1. Focus_mod Module

First, we downsample the original image (640 × 640 × 3) to reduce the calculation of spatial information, then form a 320 × 320 × 16 feature map through convolution, and reduce the loss of image information caused by the downsampling. Next, we perform 16 convolution kernels with 3 × 3 convolutions to obtain the feature map of complete information, implement MaxPooling again to reduce the layer size, expand the perceptual field, pool to form a feature map of 320 × 320 × 16, and finally combine the residuals and output a 320 × 320 × 32 feature map. Pooling removes redundant information, compresses features, simplifies the network complexity, reduces computation, reduces memory consumption, and makes the smoke feature layer more obvious. Compared with the original focus module, the parameters of the improved Focus_mod module are reduced by 6 times, and the calculation amount is reduced by 7 times, as shown in Figure 1.

#### 3.2.2. GBN (Ghost Bottleneck) Module

GhostNet proposes an innovative Ghost module that generates more feature maps through cheap operations. This new basic unit of the neural network successfully achieves more feature maps with fewer parameters and computations. The implementation of this module is divided into two parts. First, GhostNet uses a normal convolutional calculation to obtain feature maps with fewer channels, then uses a cheap operation to obtain more feature maps, and finally concatenates different feature maps together and combines them into a new output, as shown in Figure 2.

In GhostNet, the Ghost bottleneck module is divided into two types according to the stride. The Ghost bottleneck module structure when stride = 1 is modeled on ordinary residuals and is composed of two Ghost modules. The first module acts as an extension layer to increase the number of channels. The second module reduces the number of channels to match the shortcut path and then uses the shortcut to connect the inputs and outputs of these two Ghost modules. The Ghost bottleneck module when stride = 2 has the layout of the standard bottleneck structure and maintains the structural characteristics when stride = 1. By learning from the experience of the linear bottleneck module of MobileNetv2, an intermediate block is added in the middle of the stride = 1 structure. For a lightweight two-dimensional depthwise convolution, the amount of computation is reduced. This method draws on the experience of MobileNetv2. During the design process of the module and when the ReLU activation function is not used after the second Ghost module, the other layers use batch normalization (BN) and the ReLU nonactivation function after each layer. The structure design of the Ghost bottleneck is shown in Figure 3.

#### 3.2.3. Attention Mechanism

The convolutional block attention module (CBAM) is a lightweight convolutional attention module that combines channel and spatial attention mechanism modules [61]. CBAM includes two sub-modules, the channel attention module (CAM) and the spatial attention module (SAM), which perform channel and spatial attention, respectively. This not only saves parameters and computing power but also ensures that it can be integrated into the existing network architecture as a plug-and-play module. CAM is an adjustment to the structure of the SE module. Based on the SE module, a global maximum pooling operation is added to the CAM. CAM compresses the feature map into a one-dimensional vector in the spatial dimension, uses global average pooling and global maximum pooling to aggregate the feature information of the spatial map, and performs an element-by-element sum operation on the results by sharing the fully connected layer. The structure setting of the double pooling operation can make the extracted high-level features richer and provide more detailed information. SAM performs the concatenating operation on the result of the CAM operation based on the channel and performs single-channel dimensionality reduction through convolution. Similar to CAM, SAM adopts a double pooling operation. CBAM is similar to the SE module. The module structure mostly uses a 1 × 1 convolution to operate and completes the information extraction of the feature map through the entire channel dimension of the SAM, as shown in Figure 4.

### 3.3. Lightweight YOLOv5

Figure 5 shows the lightweight YOLOv5 network structure. Based on the YOLOv5s framework, the main improvements involve the two parts of backbone and neck. Combined with the introduction in Section 3.2, the overall structure of the improved lightweight network in this paper can be obtained. The multiscale output of the traditional model is output by the bottleneck module, and the modified multiscale output of the improved model is output by concatenating the two characteristic diagrams.

Table 1 shows the comparison between the parameter quantities of different sub-modules and the calculation quantities of traditional YOLOv5 sub-modules (focus, Conv, and CSP). The number of parameters and calculations of Focus_mod and GBN are significantly reduced. The parameter quantity of the Focus_mod module is 232, and the calculation quantity is 27.85 M. The parameter quantity of the GBN module is 317, and the calculation quantity is 136.4 M.

Table 2 shows the important parameters of the lightweight network model. GBN modules are used in the backbone network and head portion, and the Focus_mod and CBAM attention mechanisms are used in the backbone network portion.

### 3.4. Loss Function

The loss function of the target detection task consists of classification loss and bounding box regression loss. IoU and its improved algorithm are the most used in the bounding box regression loss. The full name of the IoU algorithm is the intersection over union, which is obtained by calculating the ratio of the intersection and union of the predicted box and ground-truth box, that is, IoU(*A*, *B*) = (*A*∩*B*)/(*A*∪*B*), where A is the prediction box and B is the ground-truth box. IoU can be used as a distance; then, Loss_IoU = 1 − IoU. The advantage of IoU is that it can reflect the detection effect of the prediction box and ground-truth box. This paper takes CIoU as the loss function of the depth convolutional model, and the specific formula is as follows:

(1) $$\begin{array}{c} \text{IoU}=\text{IoU}-\left(\frac{p^{2}\left(b,b^{gt}\right)}{c^{2}}+\alpha v\right),\\ \text{Loss}=1-\text{IoU}+\frac{p^{2}\left(b,b^{gt}\right)}{c^{2}}+\alpha v,\\ v=\frac{4}{\pi^{2}}{\left(\arctan\frac{w^{gt}}{\pi^{gt}}-\arctan\frac{w}{h}\right)}^{2},\\ \alpha =\frac{v}{\left(1-\text{IoU}\right)+v}, \end{array}$$

where *b* and *b*^*gt*^ represent the center points of prediction Box *B* and ground-truth Box *B*^*gt*^, respectively; *c* represents the square of the diagonal length of the minimum bounding Box *C*; *p* represents the calculation of the Euclidean distance between the two center points; *α* is the weight parameter; and *v* is used to measure the similarity of the aspect ratio.

## 4. Experimental Results

### 4.1. Experimental Data and Environment

There is currently no authoritative dataset similar to ImageNet for smoke detection. The dataset used in this paper comes from the dataset published by the Fire Monitoring Technology Laboratory [62] and some network images, including a total of 4829 real smoke images. The sample images are shown in Figure 6. The smoke dataset covers the smoke pictures collected in different scenarios, including indoor monitoring, outdoor monitoring, field monitoring, field monitoring tower, drone shooting, and network pictures. The smoke and background of some images are confusing to some extent. At the same time, we collected many nonsmog background images as negative samples and divided the smoke dataset into a training set and a test set at a ratio of 7 : 3.

The experimental environment in this paper is the operating system Windows 10, graphics card NVIDIA GeForce RTX3070, memory 16G, processor Intel(R) i7-11700k, software environment CUDA11.4, and PyTorch 1.8.1.

### 4.2. Evaluation Standard

In this paper, the precision rate, recall rate, average precision (AP), and mean average precision (mAP@0.5) are used as model accuracy evaluation indicators, where AP represents the area under the PR curve, and mAP@0.5 represents the average AP of all categories when IOU is set to 0.5. The specific formula is as follows:

(2) $$\begin{array}{c} P=\frac{\text{TP}}{\text{TP}+\text{FP}},\\ R=\frac{\text{TP}}{\text{TP}+\text{FN}},\\ AP=\int_{0}^{1}P\text{d}R,\\ mAP=\frac{{\sum_{i=1}^{N}AP}_{i}}{N}, \end{array}$$

where TP is the number of correctly classified bounding boxes that are predicted, the bounding box coordinates are correct, FN is the number of all unpredicted bounding boxes, and FP is the number of predicted bounding boxes that are misclassified or whose bounding box coordinates are not up to standard.

### 4.3. Experimental Results

In the network model training phase, the iteration batch size was set to 32, the decay coefficient was 0.0005, the initial learning rate was 0.001, and the total number of iterations was 300.

In order to verify the performance of the loss function, the paper uses Alpha-IoU [63] as a comparative experiment and uses CIoU as the benchmark loss function, setting alpha values of 1, 2, and 3, respectively. Among them, alpha = 1 corresponds to the method proposed in the paper.  Figure 7 shows the loss function curves corresponding to different alpha values. It can be seen from the figure that the overall performance of the method proposed in the paper is better. When alpha = 2 or 3, the detection curve has obvious fluctuations in the early stage. This means that alpha is invalid for smoke detection when the value is high.

To verify the overall performance of the proposed method, the paper gives the following comparison algorithms:

1. YOLOv5s : YOLOv5s model without optimization.
2. YOLOv5s + Ghost: modify the focus structure to Focus_mod, and all the computing modules of the backbone network use the GhostNet module.
3. YOLOv5s + Ghost + CBAM: modify the head layer, modify the CSP module to the Ghost bottleneck, and add the CBAM module.
4. YOLOv5s-Lightweight: modify the stride = 2 of the first Ghost bottleneck of the backbone network based on the previous network.

In addition, the traditional multiscale output of YOLOv5s is output after the CSP module directly extracts features, and the lightweight network model is modified to CONCAT to connect dual feature maps for the output.  Table 3 shows the parameters and floating-point calculation of the different algorithms. The parameter of the lightweight network model is only 2.75 M, and the floating-point calculation is 2.56 G, which is approximately 38% of the YOLOv5s parameter (7.25 M) and 15% of floating-point computation (16.86 G).  Figure 8 shows the precision, recall, and mAP@0.5 curves of the four models. It can be seen from the figure that the accuracy of the lightweight network model is slightly better than that of the other models, the detection speed is the fastest, and the number of parameters is the lowest.

Figure 9 shows the detection results of the lightweight network model in different scenarios (including indoor and outdoor, wild, etc.). It can be seen from the figure that the lightweight network model can accurately identify smoke targets in different scenarios. In addition, we use the deep network inference engine MNN as the framework to conduct unquantified tests on smoke images on a single-core Intel i7. The traditional YOLOv5s network model needs 140 ms, while the lightweight network model only needs 60 ms, which further improves the inference speed, reaching requirements for engineering applications.

## 5. Conclusion

To solve the problem of the smoke detection algorithm with large weight parameters and slow device reasoning speed, this paper proposes a lightweight smoke detection model based on GhostNet and CBAM. The model uses Ghost convolution instead of general convolution to improve the detection speed, uses Ghost bottleneck to replace the CSP structure in the original YOLOv5 to reduce model parameters, and increases the CBAM attention mechanism. Finally, CIoU is used as the loss function to improve the detection accuracy. Compared with the benchmark YOLOv5s model, the parameter amount and calculation amount of the improved model are significantly improved, the mAP is slightly better than that of the benchmark model, and the detection speed meets the requirements of engineering applications. The paper strikes a balance between the model accuracy and speed, optimizes the YOLOv5 model reasonably, realizes model compression, speeds up inference without reducing model accuracy, and greatly reduces the dependence on the hardware environment. At present, we have completed the development of the prototype. In the future, we will complete the quantitative processing and deployment of the model on the mobile terminal and further apply it to the field to realize real-time smoke detection.

## Figures and Tables

**Figure 1:** Focus_mod module.

**Figure 2:** Ghost module.

**Figure 3:** Ghost bottleneck module.

**Figure 4:** CBAM module.

**Figure 5:** Lightweight network model.

**Figure 6:** Sample images from the dataset.

**Figure 7:** Performance curves of different loss functions.

**Figure 8:** Performance detection curves of different models. (a) mAP@0.5. (b) Precision. (c) Recall.

**Figure 9:** Detection results with the lightweight network model.

**Table 1:** Parameters and calculations of the sub-modules.

Module	Parameters	FLOPs/M
Focus	1760	181.86
Focus_mod	232	27.85
Conv	464	196.61
CBAM	594	230.2
CSP	1120	481.69
GBN	317	136.4

**Table 2:** Overall architecture of lightweight network model.

Input	Operator	Conv	Stride	SE
640 ✕ 640 ✕ 3	Focus_mod	3 ✕ 3	1	—
320 ✕320✕64	CBAM	3 ✕ 3	2	—
160 ✕160✕64	GBN	5 ✕ 5	2	1
160 ✕160✕64	Conv	3 ✕ 3	2	—
80 ✕80✕64	GBN	3 ✕ 3	1	1
40 ✕ 40 ✕ 128	Conv	3 ✕ 3	2	—
40 ✕ 40 ✕ 128	GBN	3 ✕ 3	1	—
20 ✕ 20 ✕ 256	Conv	3 ✕ 3	2	—
20 ✕ 20 ✕ 256	GBN	3 ✕ 3	1	—
20 ✕ 20 ✕ 256	SPP	1 ✕ 1	2	—
20 ✕ 20 ✕ 512	GBN	3 ✕ 3	1	1
20 ✕ 20 ✕ 256	Conv	1 ✕ 1	1	—
40 ✕ 40 ✕ 256	Upsample			—
40 ✕ 40 ✕ 256	GBN	3 ✕ 3	1	1
40 ✕ 40 ✕ 128	Conv	1 ✕ 1	1	—
80 ✕ 80 ✕ 128	Upsample			—
80 ✕ 80 ✕ 128	GBN	3 ✕ 3	1	1
40 ✕ 40 ✕ 128	Conv	3 ✕ 3	2	—
40 ✕ 40 ✕ 256	GBN	3 ✕ 3	1	1
20 ✕ 20 ✕ 512	Conv	3 ✕ 3	2	—

**Table 3:** The performance of different models.

Model	Parameters	FLOPs (G)	mAP@0.5 (%)
YOLOv5s	7255094	16.86	97.04
YOLOv5s + Ghost	4434246	8.88	97.09
YOLOv5s + Ghost + CBAM	3624520	6.28	97.23
YOLOv5s-Lightweight	2751176	2.56	97.45

## Data Availability

The data used to support the findings of this study are included within the article.
